# Effect of Comprehensive Nursing Intervention Under Internet-Based WeChat Platform Education on Postoperative Recovery of Puerperae Undergoing Cesarean Section

**DOI:** 10.1155/2022/5040461

**Published:** 2022-04-06

**Authors:** Guixiang Kong, Jinfeng Liu, Jing Jiang

**Affiliations:** ^1^Department of Obstetrics, The Second Hospital of Shandong University, Jinan 250033, Shandong, China; ^2^Department of Emergency Surgery, College of Nursing, Shandong University of Traditional Chinese Medicine, Jinan 250355, Shandong, China

## Abstract

**Objective:**

To explore the effect of comprehensive nursing intervention under internet-based WeChat platform education on postoperative recovery of puerperae undergoing cesarean section (C-section).

**Methods:**

A total of 96 patients undergoing C-section in our hospital from June 2018 to October 2021 were selected for the retrospective analysis and grouped according to the nursing intervention modes as follows: patients who received a routine nursing intervention were included in the control group, and patients who received comprehensive nursing intervention under internet-based WeChat platform education were included in the study group, with 48 cases each. After the intervention, the postoperative recovery of puerperae undergoing C-section and obstetrics nursing quality were scientifically assessed.

**Results:**

No statistical differences in general data between the two groups were observed (*P* > 0.05). Compared with the control group, patients in the study group had obviously earlier initial time of lactation (*P* < 0.05), significantly higher breast milk amount within 48 h after delivery (*P* < 0.05), significantly earlier spontaneous urination time, anal exhaust time and off-bed activity time (*P* < 0.05), obviously better mastery of health knowledge (*P* < 0.05), and, in terms of SCL-90, remarkably lower total score, average total positive score, and the number of positive items and scores in dimensions, such as somatization, obsessive-compulsive, depression, anxiety, interpersonal sensibility, anger-hostility, phobic-anxiety, and paranoid ideation (*P* < 0.05). At discharge, 3 months, and 6 months of follow-up, patients in the study group obtained significantly higher scores on quality of life than the control group (*P* < 0.05).

**Conclusion:**

In the nursing of puerperae undergoing C-section, comprehensive nursing intervention measures based on the internet-based WeChat platform education can effectively improve the early lactation, mastery of health knowledge, and adverse emotions of puerpera and promote their postoperative recovery.

## 1. Introduction

Cesarean section (C-section) is one of the common procedures in obstetrics, and, with the development of modern medicine and continuous improvement in anesthesia, suture, infection control, and other technologies, it has become an important means of saving maternal and perinatal lives. However, as a kind of surgical operation, C-section has corresponding risks, and surgical trauma and postoperative comorbidities are the risk factors that lead to physical and mental injuries in the mother and seriously affect maternal postoperative recovery [1–4]. At the same time, social progress has also largely changed the perception of life and incrementally increased people's demands for health. Therefore, the way to promote the effect of postoperative rehabilitation and the quality of life of women who have undergone C-section has become a hot topic and a focus of clinical research. Since the introduction of the comprehensive nursing model with the tenet of “psychosomatic medicine” in our department, it has been applied to the care of puerperae undergoing C-section in the hope of providing care to the patients somatically and further promoting the psychological recovery of the patients, and, in turn, benefiting the body recovery to some extent. In recent years, more internet-based means have been used for preaching pregnancy knowledge, of which WeChat is favored by young people because of its simple operation, fast response, low cost, and least restriction [5–7]. To further improve the nursing quality and efficiency of puerperae undergoing C-section, our hospital combined the nursing process with the internet-based WeChat platform, in the hope of promoting maternal postoperative rehabilitation and improving the prognostic quality of life. Therefore, this paper will explore the impact of comprehensive nursing intervention under internet-based WeChat platform education on the postoperative rehabilitation of puerperae undergoing C-section.

## 2. Study Methods

### 2.1. Case Screening

According to the objective and plan of the study, the inclusion criteria for the patients were as follows: ① the patients were primipara with a single fetus, ② the patients met the surgical indications of C-section, ③ the patients did not have operation history, ④ the patients did not have severe organ function impairment or disorders, ⑤ the patients and their family members understood the study, and their consent was obtained for this study to review their clinical case data for analysis. The exclusion criteria were as follows: ① the patients were complicated with other severe organic diseases or malignancies, ② the patients had a cognitive disorder, communication disorder, or limb activity disorder, ③ the patients were complicated with extremely unstable underlying diseases, ④ the patients were unable to cooperate with the education on the internet-based WeChat platform or refused to receive follow-up, and ⑤ the patients went missing during the study. A total of 96 patients undergoing C-section in our hospital from June 2018 to October 2021 were selected for the retrospective analysis.

### 2.2. Grouping

According to the nursing intervention models conducted on the enrolled patients, those who accepted the routine nursing intervention were included in the control group, and those who received the comprehensive nursing intervention based on the internet WeChat platform education were included in the study group, with 48 cases each. The study met the World Medical Association Declaration of Helsinki (2013) [8].

### 2.3. Methods

Conventional nursing interventions, such as closely monitoring the perioperative changes of vital signs, uterine contraction, and vaginal bleeding in puerperae, conducting the administration of antibiotics according to the medical advice to prevent infection, providing routine life nursing, diet nursing, and drug nursing after operation, informing the puerperae to join the health education at fixed time and location every week by sticking the lecture notice sheet in the clinic, and informing the patients of their physical condition, relevant precautions, etc., were done by face-to-face interview.

The comprehensive nursing intervention based on the internet-based WeChat platform education was conducted with the following steps: (1) a WeChat education nursing group was established with the chief nurse being the group leader and the head nurse being the deputy group leader, and according to the nursing demands of puerperae undergoing C-section, the following posts were set: ① responsible for collecting patients' relevant data, including basic data, lecture content organization, nursing demands, and satisfaction investigation, ② responsible for designing the lecture form and contents suitable for WeChat platform health education, ③ responsible for editing the relevant health knowledge of WeChat education and timely updating in the WeChat platform, and ④ responsible for performing targeted communication with patients and their family members in the WeChat platform and timely answering patients' questions. (2) The nursing group leader conducted training for group members on relevant knowledge of obstetrical diseases, nursing for pregnant women, and recovery after C-section via various forms, including WeChat group and department lectures [9–11]. (3) Attention was paid to psychiatric nursing and enhancing the strength of health education. C-section, an open surgery, is necessary during delivery in case of situations, such as fetal distress, delay in labor course, and an abnormally large fetus or malposition of the fetus. Hence, patients tend to have great mental stress accompanied by anxiety, and therefore, the nursing personnel should pay special attention, keep a kind attitude, and be patient, so that the puerperae can clearly understand the treatment measures, prognosis, and enhance their confidence. The nursing personnel should also give certain psychological guidance to patients' family members for them to obtain emotional and social support as much as possible while reducing stress. After the operation, health knowledge related to infants and lactation period should be given to the patients through the WeChat platform, and a postoperative recovery plan has to be established for them. (4) Focus on rehabilitation guidance and enhancing patients' confidence in fighting the disease. After C-section, patients' movement will be constrained, and they feel pain from the operative wound. Hence, most patients are reluctant to do off-bed activities, and their prognostic recovery will be affected. Aiming at this situation, the nursing personnel should reasonably evaluate patients' condition and give corresponding guidance to enhance their awareness of self-care and confidence in recovery [12–14]. (5) In addition, offline and online pain care, diet guidance, hygiene care, breastfeeding nursing, etc., should be performed on patients after C-section to promote clinical nursing quality and postoperative recovery. (6) Steps for implementing the WeChat platform: the nursing personnel taught the pregnant women the relevant knowledge of obstetric diseases, nursing during pregnancy, and precautions after C-section and set up their own WeChat platform or official account. The puerperae discussed the knowledge they learned in the WeChat group, and the specific nursing personnel gave the specific standardized methods [15].

### 2.4. Observation Indexes

Patients' general data, including age, BMI, marital status, educational degree, work, gestational age, and newborn body mass, 1 min Apgar score, and 5 min Apgar score were recorded. Patients' early lactation, including initial time of lactation and 48 h lactation amount, was observed. Patients' early recovery situations after surgery, including spontaneous urination time, anal exhaust time, and off-bed activity time were recorded.

Patients' mastery of the health knowledge of gestation period, lactation period, and perioperative period of C-section was tested by written examination with a total score of 100 points, and higher scores indicated better mastery. The written examination was designed by our hospital according to the clinical investigations and by referring to the *Questionnaire on Maternal Health Knowledge* [16].

The degree of mental health of patients was assessed by Symptom Checklist-90 (SCL-90) (Cronbach'*α* coefficient of 0.801–0.923, and retest reliability of 0.633–0.746), which included 90 items, covered relatively extensive contents of psychic symptomatology involving aspects from feeling, emotion, thinking, awareness, behavior to living habits, interpersonal relationship, diet, and sleep, and reflected the mental symptoms with 10 factors, with higher scores indicating more serious symptoms. During follow-up visits, the SF-36 scale was adopted to evaluate the level of patients' quality of life, with higher scores indicating better quality of life. The SF-36 scale was developed by the Institute of Medicine, which is a universal scale to measure patients' QOL and has been generally recognized worldwide.

### 2.5. Statistical Processing

In this study, the data processing software was SPSS22.0, the picture drawing software was GraphPad Prism 7 (GraphPad Software, San Diego, USA), the types of data were enumeration data and measurement data, which were expressed by [*n*(%)] and ($\bar{x}$ ± *s*) and examined by *X*^2^ test and *t*-test, respectively, and differences were considered statistically significant at *P* < 0.05.

## 3. Results

### 3.1. General Data

Between the two groups, no significant differences in patients' general data, including age, BMI, marital status, educational degree, work, gestational age, and newborn body mass, 1 min Apgar score, and 5 min Apgar score were observed (*P* > 0.05). See Table 1.

### 3.2. Early Lactation

According to the statistical data in Table 2, patients in the study group had obviously earlier initial time of lactation (*P* < 0.05) and significantly higher breast milk amount within 48 h after delivery (*P* < 0.05) than the control group.

### 3.3. Early Recovery after Operation

Compared with the control group, patients in the study group had obviously earlier spontaneous urination time, anal exhaust time, and off-bed activity time (*P* < 0.05). See Figure 1.

### 3.4. Mastery of Health Knowledge

According to the result shown in Figure 2, the mastery of health knowledge was significantly better in the study group than in the control group (*P* < 0.05), presenting statistical significance in the between-group difference.

### 3.5. SCL-90 Scores

Compared with the control group in terms of SCL-90, the study group obtained remarkably lower total score, average total positive score, and number of positive items and scores on dimensions, such as somatization, obsessive-compulsive, depression, anxiety, interpersonal sensibility, anger-hostility, phobic-anxiety, and paranoid ideation (*P* < 0.05). See Table 3.

### 3.6. Quality of Life

At discharge, 3 months, and 6 months of follow-up, the scores on the quality of life were significantly higher in the study group than in the control group (*P* < 0.05). See Figure 3.

## 4. Discussion

A C-section is a traumatic procedure in which infants are delivered by open abdominal delivery to avoid damage to maternal or fetal life and health from vaginal production. Many women experience emotional swings during pregnancy because of great physical and mental stress, which, combined with the effect of surgery, can have an enormous negative impact on the puerperae. In addition, pain in the body and postoperative comorbidities, accompanied by negative emotions, such as anxiety, fear, and depression, severely affect postpartum lactation and recovery. Therefore, it is important to timely implement a series of nursing measures for puerperae undergoing C-section, so that they can eliminate negative emotions, ensure physical and mental health, follow the instructions proactively, and speed up postoperative rehabilitation. Modern medical research holds that the object of clinical medicine is a person who has thoughts and feelings in a certain social condition, and the connotation of health is not only the elimination of physical diseases but the pursuit of a complete physical and mental state and social resilience [17–20]. Based on the clinical nursing experience and related investigations in our hospital, comprehensive nursing measures with the concept of “psychosomatic medicine” were introduced, which regarded the patients as a whole, and no longer focused the nursing care alone on a disease with certain biological significance. Pregnant women are a special group receiving great concern from society, and today, with increasing emphasis on bearing and rearing better children, mastering the basic knowledge of gestational health, and spending uneventful pregnancy and puerperal period are the realistic needs of each family. The related survey has revealed that almost every pregnant woman and the accompanying family member have a strong learning need for the knowledge of maternal and child health, especially the primipara, who have a stronger desire for the knowledge of gestational health care, postnatal rehabilitation, and scientific parenting. In the face of social development, there are lesser on-site maternal lectures carried out in hospitals, which pregnant women can attend. Besides that, time, place, work, family, traffic, and other factors constrain health knowledge preaching, which also leads to women becoming overwhelmed when facing issues, such as delivery, C-section, postoperative rehabilitation, feeling anxious, and panic, adversely affecting their recovery after C-section [15, 21–23]. With the development of internet technology, a mobile phone has become a necessity for almost everyone, and WeChat, one of the communication software on mobile phones, is a representative of lifestyle in the new era and is a learning platform.

Comprehensive nursing mainly includes psychiatric nursing, pain care, dietary guidance, behavior restriction, postoperative hygiene nursing, and breastfeeding nursing. Among them, effective psychiatric nursing can help patients to eliminate negative emotions, build a positive mindset, and create a good psychological environment for postoperative recovery. Scientific postoperative pain care and hygiene nursing can directly develop an optimal physiological status for puerperae's physical rehabilitation and enable fast wound healing. Reasonable dietary guidance is an important measure for guaranteeing the physical health of puerperae and newborns, because diet therapy quickly nourishes the puerperae, invigorates the impaired body, promotes breast milk secretion, and helps body recovery, and it can also maintain the healthy development of newborns. The initial period after C-section is a critical period of body recovery and brings maximum physical stress for puerperae, and scientific behavior care is beneficial for uterine contraction and wound healing while preventing postoperative complications, such as ankylenteron and thrombosis. The comprehensive nursing mode that is established on the basis of the WeChat platform mainly enriches the forms and contents of comprehensive nursing with the help of the convenient, timely, and diversified WeChat platform and provides a more flexible comprehensive nursing during implementation to ensure that puerperae well-master health knowledge.

The study results showed that compared with the control group, patients in the study group had obviously an earlier initial time of lactation (*P* < 0.05) and significantly higher breast milk amount within 48 h after delivery (*P* < 0.05), which was consistent with the report by Sakki Kwame et al. [24] Between the two groups, patients in the study group had obviously an earlier spontaneous urination time, anal exhaust time, off-bed activity time (*P* < 0.05), better mastery of health knowledge (*P* < 0.05), obviously lower SCL-90 scores (*P* < 0.05), and significantly higher scores on quality of life at discharge, 3 months, and 6 months of follow-up (*P* < 0.05). These results indicated that sound preaching means combined with scientific nursing measures can effectively improve the physical and mental state, promote physical rehabilitation, and improve the prognostic quality of life for puerperae undergoing C-section. The reasons were as follows: (1) health preaching was also an important means for improving the level of nursing services. In this study, health knowledge related to predelivery, intrapartum, and postdelivery rehabilitation was given to the puerperae in the form of text, pictures, PPT, audio explanation, and video preaching using the WeChat platform, and by integrating online with offline, puerperae's behavior compliance with medical advice and health maintenance were improved to ensure the effect of postoperative recovery. (2) The establishment of the WeChat platform for puerperae undergoing C-section worked both ways. On the one hand, with the advantages of low cost, high flexibility, and no space limitation, WeChat greatly promoted the coverage, rate, and the extent of the spread of preaching information and enhanced the degree of adhesion between nurses and patients. On the other hand, WeChat extended the clinical nursing measures, so that the comprehensive nursing mode became more scientific and humanized with the strong promotion effect of WeChat.

In conclusion, in the nursing of puerperae undergoing C-section, comprehensive nursing intervention measures based on the internet WeChat platform preaching can effectively improve the initial lactation, promote the mastery of health knowledge, relieve adverse emotions, accelerate postoperative recovery, and upgrade the prognostic quality of life for puerperae. In addition, considering the limited study cost, only 48 patients were included in the study. Hence, the sample size was small, and deep research with a large sample size is still required. Although effective, the combination of the WeChat platform and clinical nursing is still in the phase of ongoing exploration, presenting a very high potential value to be extended. Therefore, the potential value of reducing the incidence rate of C-section with the help of internet-based WeChat platform preaching can be actively explored in the future.

## Figures and Tables

**Figure 1:** Comparison of puerperae's early recovery after operation between the two groups ($\bar{x}$ ± *s*). Note: the horizontal axis indicated the evaluation dimensions, and the vertical axis indicated the time (h). The spontaneous urination time, anal exhaust time, and off-bed activity time of the control group were (4.66 ± 0.64), (8.57 ± 1.01), and (16.63 ± 3.18), respectively. The spontaneous urination time, anal exhaust time, and off-bed activity time of the study group were (2.28 ± 0.43), (6.05 ± 0.87), and (12.08 ± 2.56), respectively. ^*∗*^indicated significant difference in spontaneous urination time between the two groups (*t* = 21.386, *P* < 0.001). ^*∗∗*^indicated significant difference in the anal exhaust time between the two groups (*t* = 13.097, *P* < 0.001). ^*∗∗∗*^indicated significant difference in off-bed activity time between the two groups (*t* = 7.722, *P* < 0.001).

**Figure 2:** Comparison of scores on mastery of health knowledge of puerperae between the two groups ($\bar{x}$ ± *s*). Note: the horizontal axis indicated the evaluation dimension, and the vertical axis indicated the score. The score on the mastery of health knowledge of the control group was (90.12 ± 4.85). The score on the mastery of health knowledge of the study group was (97.38 ± 2.55). ^*∗*^indicated significant difference in scores on the mastery of health knowledge between the two groups (*t* = 9.179, *P* < 0.001).

**Figure 3:** Comparison of scores on puerperae's quality of life between the two groups ($\bar{x}$ ± *s*). Note: the horizontal axis indicated the time points, and the vertical axis indicated the score. At discharge, 3 months, and 6 months of follow-up, the scores on the quality of life of the control group were (40.07 ± 9.22), (55.64 ± 10.62), and (70.55 ± 11.05), respectively. At discharge, 3 months, and 6 months of follow-up, the scores on the quality of life of the study group were (47.86 ± 8.91), (64.45 ± 8.22), and (76.88 ± 10.54), respectively. ^*∗*^indicates significant difference in scores on the quality of life at discharge between the two groups (*t* = 4.209, *P* < 0.001). ^*∗∗*^indicates significant difference in scores on the quality of life at 3 months of follow-up between the two groups (*t* = 4.545, *P* < 0.001). ^*∗∗∗*^indicates significant difference in scores on the quality of life at 6 months of follow-up between the two groups (*t* = 2.872, *P*=0.005).

**Table 1:** Comparison of patients' general data between the two groups (*n* = 48).

Observation indicator	Control group	Study group	*X* ^2^/*t*	*P*
Age (years)	27.59 ± 2.16	28.12 ± 2.23	1.183	0.240
BMI (kg/m^2^)	23.71 ± 3.25	23.85 ± 3.11	0.216	0.830
Marital status			0.300	0.584
Married	39 (81.25)	41 (85.42)		
Unmarried	9 (18.75)	7 (14.58)		
*Educational degree*				
Junior high school and below	6 (12.5)	5 (10.42)	0.103	0.749
Senior high school	25 (52.08)	24 (50)	0.042	0.838
Above senior high school	17 (35.42)	19 (39.58)	0.178	0.673
Work			0.178	0.673
Manual labor	17 (35.42)	19 (39.58)		
Brain work	31 (64.58)	29 (60.42)		
Gestational age (weeks)	38.25 ± 1.74	38.19 ± 1.71	0.170	0.865
*New-born*				
Body mass (kg)	3.59 ± 1.10	3.69 ± 1.09	0.447	0.656
1 min Apgar score	7.56 ± 1.43	7.67 ± 1.35	0.388	0.699
5 min Apgar score	8.43 ± 1.26	8.51 ± 1.30	0.306	0.760

**Table 2:** Comparison of puerperae's lactation between the two groups ($\bar{x}$ ± *s*).

Group	*n*	Initial time of lactation (h)	Breast milk amount within 48 h after delivery (ml)
Control	48	38.16 ± 4.83	370.15 ± 24.08
Study	48	28.76 ± 3.40	429.96 ± 42.19
*t*		11.026	8.530
*P*		<0.001	<0.001

**Table 3:** Comparison of puerperae's SCL-90 scores between the two groups ($\bar{x}$ ± *s*).

Evaluation dimension	Control group	Study group	*t*	*P*
Total score	134.22 ± 19.83	115.96 ± 15.23	5.060	<0.001
Number of positive items	27.18 ± 9.32	18.15 ± 8.02	5.088	<0.001
Average total positive score	2.14 ± 0.40	1.12 ± 0.43	12.033	<0.001
Somatization	2.07 ± 0.42	1.33 ± 0.44	10.066	<0.001
Obsessive-compulsive	2.31 ± 0.35	1.35 ± 0.37	13.059	<0.001
Depression	2.27 ± 0.23	1.34 ± 0.25	18.967	<0.001
Anxiety	2.38 ± 0.22	1.36 ± 0.26	20.749	<0.001
Interpersonal sensibility	2.29 ± 0.37	1.36 ± 0.35	12.651	<0.001
Anger-hostility	2.01 ± 0.29	1.01 ± 0.33	15.770	<0.001
Phobic-anxiety	1.45 ± 0.28	1.04 ± 0.22	7.977	<0.001
Paranoid ideation	1.55 ± 0.30	1.09 ± 0.32	7.266	<0.001
Psychoticism	1.55 ± 0.23	1.08 ± 0.16	11.622	<0.001

## Data Availability

Data to support the findings of this study are available on reasonable request from the corresponding author.
